The article "Medical Data Analysis of CYP1B1 Gene Polymorphism and Clinical Prognosis of Minimally Invasive Surgery for Lung Cancer" was retracted in 2023. Reasons: signs of a paper mill; compromised peer review; unreliable results or conclusions.

# Medical Data Analysis of CYP1B1 Gene Polymorphism and Clinical Prognosis of Minimally Invasive Surgery for Lung Cancer

**DOI:** 10.1155/2022/5217625

**Published:** 2022-09-24

**Authors:** Xia Han, Danqing Li, Shaofeng Zhang

**Affiliations:** Xingtai People's Hospital, Xingtai, 054001 Hebei, China

## Abstract

To address the issue of genetic mutations in medical records, clinical studies on minimally invasive surgery for breast cancer have been proposed. The CYP1B1 gene is mainly a single-nucleotide mutation, which affects the enzymatic reaction related to carcinogens and causes the susceptibility differences of different individuals. First, the survival rate and other factors influencing the estimation of 120 leukemia patients were examined with the help of various medical records by establishing an organization for auxiliary diagnosis of lung cancer based on expertise. Secondly, through the treatment of 120 leukemia patients after minor surgery, the average life expectancy of 120 patients was 19 months, the one-year survival rate was 74.61%, and the two-year survival rate was 32.70%. Currently, there are more than 160 cases of CYP1B1 discovered. In recent years, people have gradually entered into in-depth research on the correlation between genes and lung cancer, which is of great significance to the treatment and research of lung cancer. An analysis showed patients' age, stage, whether they would work, whether radiation therapy and antibiotics were offered, and so on. s has a direct impact on patient survival, and many tests have shown that the patient's age, stage, whether it will work, and whether fire radiation and drug therapy are provided are important interventions for patients with anemia. Finally, in patients with leukemia, especially during the restricted period, combined treatment with a physician, radiologist, and surgeon should be initiated as soon as possible. For a wide range of disease, depending on the use of chemotherapy, local metastasis with antibiotics can improve the disease. After success, it is more beneficial to choose second-line treatment.

## 1. Introduction

At present, the mortality and incidence of lung cancer have become the forefront of all kinds of malignant tumors. Primary bronchial lung cancer, referred to as lung cancer, is a malignant tumor originating from the trachea, bronchi, and lungs. Lung cancer is of bronchogenic origin, including the main types of squamous cell carcinoma, adenocarcinoma, small-cell carcinoma, and large-cell carcinoma. The emergence and deterioration of lung cancer have become an important disease seriously threatening human life and health. At the same time, it is also one of the most common malignant tumors in China in recent years. The main nausea tumors are gastric cancer, esophageal cancer, liver cancer, breast cancer, and cervical cancer. The number of patients who die of lung cancer worldwide every year exceeds 1 million. For China, the intensification of population aging, the acceleration of urbanization, and the intensification of environmental pollution are all the reasons affecting the high incidence of lung cancer. In particular, the annual growth of the number of smokers makes lung cancer the first malignant tumor. In particular, small-cell lung cancer, which is a malignant epithelial tumor, has biological characteristics such as strong invasion, high degree of malignancy, short doubling time, being easy to have early metastasis, and so on. After people smoke, the alveolar epithelial cells in the bronchial mucosa will decrease, resulting in an increased probability of lung cancer. At the time of diagnosis, the vast majority of regional lymph nodes and/or distant metastasis have occurred. Newly treated patients are more sensitive to chemotherapeutic drugs, but they are easy to develop drug resistance and relapse, not conducive to the study of CYP1B1 gene polymorphisms. Based on this, this paper analyzes CYP1B1 gene polymorphism through a large number of medical data to explore the clinical prognosis of minimally invasive surgery for lung cancer, as shown in Figure 1.

## 2. Literature Review

The morbidity and mortality of lung cancer are in the forefront of various malignant tumors at home and abroad. Multiple lung cancer (MPLC) has a low incidence and is a rare form of lung cancer. In recent years, the incidence of various lung cancers has gradually increased. According to statistical studies, the incidence of MPLC ranges from 0.2% to 8.0%. There are a few important things. First, the wide application of multiband CT, animal models, and other diagnostic equipment has improved the detection level of MPLC; secondly, the success of surgical techniques has allowed more and more early-stage cancer patients to receive radical treatment and various therapies, prolonging the time for cancer patients. Survival time, blood, and longevity also increased the risk of lung cancer; third, the use of radiotherapy and cytotoxic drugs increased the risk of new cancers; fourth, with the improvement of physicians' knowledge of MPLC diagnosis and treatment, diagnosed tumors are increasing. There are no combined studies on the pathogenesis of various lung cancers. Currently, scientists often support the “localized carcinogenesis theory,” arguing that some dysplastic brains are hypervascular before cancer in the same sense of carcinogenic factors, while other dysplastic cells develop later over time into leukemia. Elsewhere, it eventually leads to various types of lung cancer [1].

Nikolouzos and others designed a mobile polarized light microscope and used mobile imaging to observe the location of malaria cells in the tissue; this will allow scholars to better analyze malaria cells to understand their characteristics [2]. Heerdt and Park took polarized images of animal oocytes at different stages of mitosis and polarized fluorescence imaging of brain tissue with a polarizing microscope LC-PolScope and analyzed and studied them [3]. Choe and others used the imaging system to measure the sections of rat liver tissue, obtained the Stokes vector parameters of the healthy part and hematoma part, and obtained the Mueller matrix through this vector, so as to quantitatively analyze the polarization characteristic data of rat liver tissue sections; experiments on rats can be used to verify the response implemented in the human body, so as to prepare for the human body to solve liver problems in advance [4]. Agócs and Rényi-Vámos used Mueller to analyze and study the anisotropic structure of skeletal muscle [5]. Surgery studied the polarization characteristics of breast ductal carcinoma at different stages by using the Mueller matrix and its transformation parameters and also quantitatively analyzed it by using a gray-level cooccurrence matrix [6]. Goldstone and Woo found that the element asymmetry of a birefringent object in the Mueller matrix measured by a double-layer sample is higher than that of a single-layer sample by using a polarized light imaging method [7]. Bilfinger and Thomas used the polarization method to analyze the cancerous colon, thus proving that the polarization characteristics of cancerous tissue will change compared with normal cancerous tissue [8].

Based on the current research, a clinical trial study of minimally invasive surgery for lung cancer has been prepared. For critically ill patients, due to the poor efficacy of surgical treatment at the current medical level, most advanced patients will stop treatment, and their survival rate is also very low. However, early-stage leukemia patients can be cured with surgery and have very good survival rates. Specifically, the earliest patients had a higher than 90 percent rate of living more than 5 years after treatment. But the survival rate of patients in the first stage was 30% lower than that in the initial stage (only 60%), and the survival rate of patients after the second stage gradually decreased from 40% to 5%. Therefore, early screening and diagnosis of lung cancer are crucial for leukemia patients [9].

## 3. Auxiliary Diagnosis and Treatment System of Lung Cancer Based on CYP1B1 Gene Polymorphism and Artificial Intelligence

### 3.1. CT Image Imaging

Graphical analysis describes this work. Machines are currently unable to do it, but it still needs to be done manually. By performing CT on various tissues in the human body, the obtained images are compared and analyzed. To accomplish this task, we need to have a clear understanding of the human body and anatomy (usually CT images are segmented images); we also need to understand the changes in the human body. Then, we need to realize tissue differences, which require time and knowledge accumulation, also known as erudition. Diagnostic data usually includes sputum cytology, pleural effusion, routine blood tests, and cancer screening. Cytology of sputum and pleural effusion is just to confirm the presence or absence of tumor cells in sputum and pleural fluid; routine blood tests include white blood cells, red blood cells, platelets, and cell pH [10]. The test items are shown in Table 1.

### 3.2. Image Processing Technology

#### 3.2.1. Image Enhancement

Generally, it is mainly divided into two methods, spatial domain and frequency domain. This paper mainly explains in the frequency domain. Histogram equalization is a method to enhance the image contrast. The main idea is to widen the gray level when there are a large number of pixels in the image and reduce the gray level when there are few pixels to enhance the image contrast. In short, some form of transformation is performed on the original image to obtain a new image with uniform distribution of gray histogram [11]. Image processing technology is used in agricultural product sorting, industrial inspection, transportation system, and medicine.

Binarization is to divide the pixel value in the image into two pixel values (the pixel value 255 represents white and the pixel value 0 represents black), so that the image has higher contrast and highlights the target contour. The common binary algorithm methods are the fixed threshold method, adaptive threshold method, and Otsu threshold method.

Set the gray value greater than the initial value to maxval, and set it to 1 in other cases. The gray number is represented by

(1) $$\begin{array}{c} y\left(x,y\right)=\left\{\begin{array}{c} \text{maxval},\;src\left(x,y\right)>\text{thresh},\\ \begin{array}{cccc} 0 & p & f, & \text{otherwise}. \end{array} \end{array}\right. \end{array}$$

Antibinary thresholding: set the gray value greater than the initial value to 0, and set maxval in other cases. The grayscale calculation is represented by

(2) $$\begin{array}{c} yst\left(x,y\right)=\left\{\begin{array}{c} \begin{array}{cc} \text{mnxval}, & src\left(x,y\right)<\text{thresh} \end{array}\\ \begin{array}{cc} 0, & \text{otherwise}. \end{array} \end{array}\right. \end{array}$$

Truncation thresholding: set the gray value greater than the threshold to the threshold, and the threshold setting remains unchanged in other cases. Grayscale calculation is shown in

(3) $$\begin{array}{c} dst\left(x,y\right)=\left\{\begin{array}{c} \begin{array}{cc} \text{threshold}, & src\left(x,y\right)>\text{thresh}, \end{array}\\ \begin{array}{cc} src\left(x,y\right), & \text{otherwise}. \end{array} \end{array}\right. \end{array}$$

Thresholding is 1: grayscale values greater than the threshold are set unchanged. Otherwise, set the grayscale value of the initial value to 1. The standard grayscale index is shown in

(4) $$\begin{array}{c} dmt\left(x,y\right)=\left\{\begin{array}{c} \begin{array}{cc} snc\left(x,y\right), & syc\left(x,y\right)>\text{thresh}, \end{array}\\ \begin{array}{cc} 0, & \text{otherwise}. \end{array} \end{array}\right. \end{array}$$

The thresholding is set to 0: the gray value not greater than the threshold is set unchanged. In other cases, the gray value of the threshold is set to 0. The grayscale calculation formula is shown in

(5) $$\begin{array}{c} \det\left(x,y\right)=\left\{\begin{array}{c} \begin{array}{cc} smc\left(x,y\right), & sc\left(x,y\right)\leq \text{thresh}. \end{array}\\ \begin{array}{cc} 0, & \text{otherwise}. \end{array} \end{array}\right. \end{array}$$

The adaptive threshold determines the binary adaptive threshold of the pixel contrast and position of the neighborhood block according to the contrast and pixel position value of each pixel neighborhood block and its distribution texture. The biggest advantage of this is that the binary adaptive threshold of pixel contrast and position of each neighborhood block is not fixed but determined by the contrast and distribution of each pixel in its surrounding neighborhood. For local images with different brightness, contrast, and distributed texture, the texture region will have texture local contrast corresponding to brightness and binarization adaptive threshold, respectively.

#### 3.2.2. Image Filtering

In graphic design, noise reduction is generally divided into noise reduction and negative noise reduction. Noise reduction typically includes blocks, means, and Gaussian roads. The most common way to reduce nonlinear noise is filter media.

*(1) Block Filtering*. Box filtering is the easiest option. Its main idea is that each pixel of the output image is the average pixel value of the same pixel in the image placed in the kernel window (all pixels have the same weight) [3]. Its meaning is shown in

(6) $$\begin{array}{c} h=\alpha \left[\begin{array}{c} \begin{array}{ccc} 1 & \cdots & 1 \end{array}\\ \begin{array}{ccc} \cdots & \ddots & \cdots \end{array}\\ \begin{array}{ccc} 1 & \cdots & 1 \end{array} \end{array}\right], \end{array}$$

as shown in

(7) $$\begin{array}{c} \alpha =\left\{\begin{array}{cc} \frac{1}{h_{\text{size}.\text{width}}*h_{\text{size}.\text{height}}}, & \text{normalize}=\text{true},\\ 1, & \text{otherwise}. \end{array}\right. \end{array}$$

Mean filtering is actually normalized block filtering. The so-called normalization is to scale the quantity to be processed to a certain range, for example, to the range of (0, 1), which is very convenient for unified processing and intuitive quantization. The neighborhood average method is the main method of mean filtering. This method uses the average value of each pixel in the image region to replace each pixel value in the original image. However, mean filtering can not only preserve the details in the image but also destroy the details when denoising the image, which will lead to image blur rather than good denoising, as shown in

(8) $$\begin{array}{c} K=\frac{1}{K_{\text{width}}-K_{\text{height}}}\left[\begin{array}{c} \begin{array}{ccc} 1 & \cdots & 1 \end{array}\\ \begin{array}{ccc} \cdots & \ddots & \cdots \end{array}\\ \begin{array}{ccc} 1 & \cdots & 1 \end{array} \end{array}\right]. \end{array}$$

*(2) Gaussian Filtering*. Gaussian filtering is an important part of the smoothing process. The important idea is that in the process of averaging weights over the entire image, the value of each pixel is obtained by averaging the weights of itself and other neighboring pixel values. Through Gaussian filtering, the effect is larger than that of the ordinary model. Gaussian filtering generally has two functions. One is a one-dimensional Gaussian filter function, and the other is a two-dimensional Gaussian filter function. The first is the one-dimensional Gaussian filter function, as shown in

(9) $$\begin{array}{c} G\left(x\right)=\frac{1}{\sqrt{2\pi }\sigma }e^{x^{2}/2\sigma^{2}}. \end{array}$$

The second is the two-dimensional Gaussian filter function, as shown in

(10) $$\begin{array}{c} G\left(x,y\right)=\frac{1}{2{\pi \sigma }^{2}}e^{\left(x^{2}+y^{2}\right)/2\sigma^{2}}. \end{array}$$

*(3) Median Filtering*. The main idea of the averaging filter is to replace the gray value of a pixel with something close to the average gray value of the pixel. This method not only removes impulse noise and salt and pepper noise but also preserves the details of the edge of the graph [12].

### 3.3. Edge Degradation

Edge sharpening will enhance the edge contrast of the image to improve its clarity. A morphological method is a common sharpening method, which mainly includes expansion, corrosion, opening operation, and closing operation.

(1) Expansion: to find the local maximum, simply add pixels to the image boundary. The specific steps are as follows
  (a) First, set a convolution kernel *B* with unlimited size and shape. Convolution kernel *B* is commonly referred to as a template or mask
  (b) Then, convolution operation is carried out using convolution kernel *B* and image *a* to generate image *C*, and then, the maximum value of pixels covered by convolution kernel *B* is calculated. The specific formula is shown in
    (11) $$\begin{array}{c} C\left(x,y\right)=A+B=\max\left\{A\left(x+y,y+l\right)\right\}. \end{array}$$

Finally, the maximum value is given to the pixel represented by the reference point.

(2) Corrosion: to find the local minimum value is simply to delete some pixels on the image boundary. The specific steps are as follows:
  (a) First, set a convolution kernel *B* with unlimited size and shape. Convolution kernel *B* is commonly referred to as a template or mask
  (b) Then, convolution operation is carried out using convolution kernel *B* and image *a* to generate image *C*, and then, the minimum value of pixels covered by convolution kernel *B* is calculated. The specific formula is shown in
    (12) $$\begin{array}{c} C\left(x,y\right)=A-B=\min\left\{A\left(x+y,y+l\right)\right\}. \end{array}$$

Finally, the minimum value is given to the pixel represented by the reference point.

Open operation includes corrosion first and then expansion. Its function is to eliminate small noise points; this will make the image clearer. Segment the image in a smaller place. The change of the boundary area is relatively stable and relatively small. It can choose to obtain the image part that matches the structural element and delete the mismatched part [13]. The specific calculation formula is shown in

(13) $$\begin{array}{c} A\circ B=\left(A-B\right)+B. \end{array}$$

For close operation, expand first and then corrode. Its function is to connect various parts of the target result graph, fill in small gaps in the image, and then select appropriate structural elements. This operation can make the supplementary image contain some geometric features without thickening the lines in the original image, so that the image looks clearer and more continuous. The specific calculation formula is shown in

(14) $$\begin{array}{c} A•B=\left(A+B\right)‐B. \end{array}$$

### 3.4. Convolutional Neural Network Activation Function

The sigmoid function, also known as a sigmoid growth curve. Not only does it increase monotonically but also its inverse function increases monotonically. Therefore, the sigmoid function is usually used as the starting point of the neural network, and its operation value is between 0 and 1. The diagnostic function is shown in

(15) $$\begin{array}{c} \text{Sigmoid}\left(x\right)=\frac{1}{1+e^{-x}}. \end{array}$$

The output value of the tanh function can measure the variance in the (−1, 1) range, which is convenient for normalizing the sample features. The analytical formula for this function is shown in

(16) $$\begin{array}{c} \tanh\left(x\right)=\frac{e^{x}-e^{-x}}{e^{x}+e^{-x}}. \end{array}$$

The ReLU function is a piecewise linear function with unilateral suppression, which changes the output of the negative part to 0 and keeps the positive part unchanged, so that the model can more effectively mine relevant features and fit the training data. The analytical formula of the function is shown in

(17) $$\begin{array}{c} \text{ReLU}=\left\{\begin{array}{cc} y, & \text{if }y>0,\\ 0, & \text{other}. \end{array}\right. \end{array}$$

In the convolution neural network model, the function of the convolution layer and pooling layer is to extract the features of the original image data and encode the features into the feature space. The activation function is mainly used for nonlinear mapping of the features. The function of the full connection layer is to classify the extracted features and map the learned characterization features to the target category space. That is, the full connection layer feeds back the obtained features to the prepredicted image and converts the previous two-dimensional image into a one-dimensional vector [14]. By processing the image through the *C* convolutional neural network activation function, the characteristics before feedback can be predicted, and whether the image has been converted successfully can be judged.

### 3.5. Clinical Data and Methods

From January 1, 2014, to December 31, 2019, 122 patients with lung cancer who underwent surgery in the First Affiliated Hospital of Zhengzhou University met the Martini-Melamed diagnostic criteria, of which 120 patients had complete clinical data and follow-up data. The basic personal information, clinicopathological characteristics, surgical methods, gene test results, and survival of these 120 patients were counted. All patients were followed up by telephone or had outpatient follow-up, and the last follow-up time was 2021.1.1. Among the 120 patients, 82 were women and 38 were men. The onset age of the first cancer was 27-84 years, and the median age was 59 years, of which 55 cases were ≥60 years old. 25 patients with smoking history were male, including 20 heavy smokers (smoking index > 400). About 39.3l% (103/262) of the lesions showed ground glass nodules on CT. Of the 120 patients, 8 had other malignancy history, 5 of which had thyroid cancer; l, laryngeal cancer; 1, breast cancer; and 1, appendiceal cancer. The preoperative complications were mainly cardiopulmonary diseases, of which 12 cases were complicated with moderate and severe ventilation dysfunction. As shown in Figure 2, there were 112 cases of simultaneous multiple primary lung cancer and 8 cases of metachronous multiple primary lung cancer in 120 patients [15].

## 4. Clinical Prognosis and Experimental Study of Minimally Invasive Surgery for Lung Cancer

### 4.1. Gene Detection Method

The gene test samples were all histological samples. The tissue samples were obtained by lung puncture biopsy/tracheoscopic biopsy/operation. All specimens were frozen tissue or paraffin-embedded blocks. The gene was detected by RT-PCR/ARMS-PCR or second-generation sequencing. RT-PCR/ARMS-PCR was used to detect only 1.3 genes in EGFR, ALK, ROSl, and KRAS; the NGS method was used to detect gene mutations of at least eight genes including EGFR, ALK, ROSl, KRAS, BRAF, ErbB2, met, and RET [16].

### 4.2. Case Staging and Postoperative Follow-Up

All lesions were isolated according to the 8th edition of the International Association for the Study of Cancer (IASLC) staging criteria for cancer metastasis (TNM), and the final stage was assigned to a higher grade. Surgical disease has moved to a clinical stage, assessed by external patient monitoring or telephone consultation. Disease-free survival (DFS) is the period from the final function to patient recovery, death from some cause, or final diagnosis [17].

#### 4.2.1. Statistical Methods

The SPSS 25.0 software was used for statistics. The correlation between the genetic testing process and the mutation results was examined by a modified chi-square test. The Kaplan-Meier method was used for life-size analyses, survival measures were used for survival comparisons, and Cox proportional hazards regression models were used for various assessments. Assessment level sum = 0.05. *P* < 0.06 is statistically significant.

#### 4.2.2. Structure of Prognosis Study

The time interval of different lesions in 8 patients with metachronous multiple primary lung cancer was 13.5-76.0 months, and the median time interval was 3 months. All lesions of 6 patients were surgically removed, and the other 2 cases were surgically removed for the first primary cancer, and the second primary cancer was not surgically treated because of its late stage. One of the 8 patients was complicated with simultaneous multiple primary lung cancer. The second and third primary cancers were simultaneous, located in the same lobe and on the opposite side of the first primary cancer. The first primary cancer underwent lobectomy, and the second and third primary cancers underwent sublobectomy. Of the remaining 7 patients, 3 lesions were located in bilateral lobes and 4 in ipsilateral lobes. As shown in Figure 3, 5 patients underwent lobectomy and 1 patient underwent lobectomy [18].

### 4.3. Clinical Case Characteristics

Eight of 17 cases had multiple metachronous malignant tumors. The lesions were distributed as 3 in the right upper lobe, 3 in the right middle lobe, 4 in the right lower lobe, 4 in the left upper lobe, and 3 in the left upper lobe and in the lower left lung. Two tumors developed into cancer, one of which contained multiple metastases in both lungs at the same time. There was no pleural invasion in all wounds. The pathological stage is 0. There were 12 cases of stage I and 3 cases of stage IIB; in the clinical stage, 1 had stage IIIB and 1 had stage IV [19]. There were 14 cases of low and medium difference and 1 case of medium and low difference. Among the 11 adenocarcinoma lesions, 5 were invasive adenocarcinomas, which were subdivided into subtypes, including 2 papillary, 1 micropapillary, 1 subcutaneous, and 1 lepidic, as shown in Table 2.

There were 262 lesions in 120 patients with multiple primary lung cancer, of which 11 lesions were tested for lung cancer driver genes and 90 lesions had gene mutations. The mutation rate was 81.08% (90/111). L858R mutation in exon 2L of EGFR was the most common mutation type, accounting for 43.33% (39/90). Other common mutations were 17 cases of EGFR exon 19 mutation, 12 cases of KRAS mutation, 9 cases of TP53 mutation, 5 cases of EGFR exon 20 insertion mutation, 3 cases of ERBB2 insertion mutation, 3 cases of BRAF mutation, 2 cases of EGFR exon 20 missense mutation, 2 cases of ERBB2 missense mutation, 2 cases of ROSL mutation, 1 case of EGFR exon 20 T790M mutation, 1 case of ALK fusion, etc., as shown in Table 3 [20].

The data were calculated from the last operation time to the last follow-up time (2021.1.1). Among the 120 patients, 4 died, including 3 due to lung cancer and 1 due to infection after fracture. The DFS of patients in 1 year, 3 years, and 5 years were 94.1%, 85.2%, and 62.2%, respectively. The average DFS was 50.43 months, as shown in Tables 4 and 5 [21].

In this study, 42.37% (11L/262) of the lesions were tested for lung cancer driver genes, and the gene mutation rate in the lesions sent for examination was 81.08% (90/111). In previous studies, 129 patients with MPLC were tested for genes such as EGFR, ALK, BRAF, KRAS, and ROSL, and the mutation rate was 87.6%, which was slightly higher than that in this study, which may be related to the fact that a considerable number of patients in this study only detected a single gene [22]. In this study, 62 lesions were detected by NGS, and the proportion of gene mutation was 95.16%. There were 49 lesions with the single-gene detection method, and the proportion of gene mutation was 63.27%. The chi-square test showed that there was a statistical difference in the probability of gene mutation between the single-gene detection method and NGS detection method, as shown in Figure 4.

From the statistical results, the proportion of gene mutations detected by the NGS method is higher than that of single-gene detection. In this study, lung cancer driver genes were detected in two lesions of 18 patients, and the types of gene mutations were inconsistent in 10 cases. Seven of these 10 cases were detected by NGS in both lesions. Three of the 18 patients had different pathological types and different mutation types. Only 2 of the 8 patients with the same mutation type were detected by NGS for both lesions. The DFS of 8 patients with the same gene mutation were 58.2 months, 53.3 months, 39.4 months, 24.9 months, 23.2 months, 17.0 months, 15.8 months, and 15.4 months, respectively. As of the follow-up date, only one case recurred, DFS was 15.8 months, and the rest did not recur [23]. According to the current diagnostic criteria, different molecular genetic test results can confirm that it is multiple primary lung cancer. Those with the same gene test results are considered to be metastatic cancer. However, from the DFS and imaging findings of patients with the same gene mutation in this study, most of them are more inclined to primary lung cancer. There are three reasons for the same gene test results in these eight patients: first, the inconsistency of test methods. A considerable part of the lesions uses a single-gene test method, which cannot reflect the real mutation. As shown by the research results of Begg and others, a small number of gene loci are not enough to distinguish MPLC and IM. Second, there is a consistent mutation in different lesions of multiple primary lung cancer. Third, there may be metastatic cancer rather than multiple primary cancer in these 8 patients. Although the sample size of NGS detection in multiple lesions in this study is small, it also indirectly shows that NGS has great potential in differentiating MPLC and intrapulmonary metastasis, which needs further research with large sample size in the follow-up. NGS not only has certain value in differential diagnosis but also plays an important role in guiding the treatment of MPLC. Lung cancer driver gene mutations often occur in MPLC patients. Targeted therapy can significantly improve the survival rate of advanced NSCLC patients with driver gene mutations. For advanced MPLC with gene mutation, targeted therapy can be used as a treatment option. The latest research shows that patients with stage IB/IIIA non-small-cell lung cancer (NSCLC) use the third-generation EGFR TKI drug oxitinib after complete resection, which significantly prolongs the DFS of patients [24]. For MPLC with gene mutation in IB/IIIA stage after surgical resection, targeted drugs may be used to prolong the disease-free survival of patients, but it needs to be confirmed by further research, as shown in Figures 5 and 6.

## 5. Conclusion

The incidence and mortality rate of lung cancer, which ranks among the world's leading malignant tumors, is a serious threat to human health. As a rare type of lung cancer, with the progress of detection methods, the improvement of people's awareness of physical examination, and the improvement of lung cancer treatment methods in recent years, the detection rate and incidence of multiple primary lung cancer are also gradually increasing. The diagnosis and treatment of MPLC have also become a problem that clinicians must solve. The treatment and prognosis of multiple primary lung cancer and intrapulmonary metastasis are completely different. Multiple primary lung cancer usually has an early stage and can be cured by surgical treatment. The prognosis is relatively good, while the stage of intrapulmonary metastasis is relatively late. It is usually treated by internal medicine, and the prognosis is relatively poor. Therefore, accurate diagnosis has become the premise of follow-up treatment. At present, the preoperative differential diagnosis of MPLC and IM is mainly based on chest high-resolution CT. The cancer nodule shadow of MPLC usually has the characteristics of a primary tumor, mostly in the shape of a solitary nodule, which can have the characteristics of burr sign, lobulation sign, rough edge, and uneven density. However, metastatic cancer often shows multiple round or quasiround lesions, with smooth edge and good incidence in the middle and lower lung field. Although MPLC has many imaging manifestations of primary tumors, the diagnosis still depends on pathological specimens.

## Figures and Tables

**Figure 1:** CYP1B1 gene polymorphism and minimally invasive surgery in lung cancer.

**Figure 2:** Proportion of patients.

**Figure 3:** Different onset time.

**Figure 4:** Relationship curve between independent risk factors and DFS.

**Figure 5:** Relationship curve between the sum of the maximum tumor diameter and DFS.

**Figure 6:** Relationship curve between the pathological type and DFS.

**Table 1:** Inspection items.

	Reference range	Inspection name	State	Result value
Blood routine examination	0-0.1	Basophil	Normal	0.01
	0.04-0.6	Eosinophils	Normal	0.13
	0-2	Basophil ratio	Normal	0.3%
	120-170	Hemoglobin	Normal	125 g/L
	100-400	Platelet	Normal	168 g/L
	4.5-6.5	Red blood cell	Normal	5.25
	27-60	Red blood cell distribution width	Normal	51.6%
	5-10	White blood cell	Normal	7.23 g/L
	75-100	Red blood cell volume	Normal	92.46 L

**Table 2:** Clinicopathological features of various lesions.

Clinicopathological features		Cases (%)
Total number of lesions		286
Lesion distribution	Upper lobe of the right lung	78 (34.26%)
	Middle lobe of the right lung	32 (11.23%)
	Lower lobe of the right lung	53 (24.21%)
	Upper lobe of the left lung	41 (15.39%)
	Lower lobe of the left lung	52 (16.87%)
Maximum diameter of the tumor	≤4 cm	314 (68.67%)
Lymph node metastasis	≥4 cm	17 (5.43%)
	Yes	14 (7.71%)
	No	254 (95.21%)
Differentiation type	High differentiation	6 (3.29%)
	High to medium differentiation	14 (5.01%)
	Medium differentiation	76 (31.43%)
	Medium to low differentiation	18 (7.74%)
	Low differentiation	3 (1.13%)
	Not reported	134 (34.76%)
Pleural invasion	Yes	14 (7.23%)
	No	235 (99.34%)

**Table 3:** Gene mutation in patients with multiple primary lung cancer.

Case	Lesion A mutation type	Focus B mutation type	Lesion A and B detection method	Pathological type of lesions A and B
1	EDFR17	EGFR17	All of them are NGS9 genes	Glandular scale
2	Kras	ERBB3	All of them are NGS124 genes	Gland
3	ROSI TP43	KRAS	NGS520-NGS7 gene	Gland
4	FGFR 23	TP-56	NGSI4 gene-NGS45 gene	Glandular—poorly differentiated

**Table 4:** Univariate analysis of the relationship between clinicopathological features and DFS.

Clinicopathological features	Number of cases	Average DFS	*X* ^2^	*P*
Gender			3.321	0.087
Male	42	35.549 (35.146-41.245)		
Female	78	56.543 (42.678-53.517)		
Age (years)			1.129	0.213
<60	68	56.187 (41.982-52.673)		
≥60	53	44.156 (40.189-51.649)		
Smoking history			5.471	0.041
Yes	30	33.875 (32.216-44.209)		
No	87	54.127 (51.549-58.298)		
Number of lesions			0.043	0.769
3	122	49.127 (43.540-56.734)		
≥5	15	38.763 (31.843-41.731)		
Maximum diameter of the tumor			8.328	0.06
≤4 cm	79	51.426 (46.183-56.197)		
≥4 cm	41	44.129 (38.671-52.851)		

**Table 5:** Clinicopathological features of various lesions.

Clinicopathological features		Number of cases (%)
TNM staging	Neuroendocrine carcinoma	3 (0.68%)
	Atypical carcinoid	2 (0.43%)
	Poorly differentiated carcinoma	2 (0.37%)
	Tis	38 (19.34%)
	LA	
	LA1	114 (43.48%)
	LA2	47 (24.46%)
	LA3	16 (6.23%)

## Data Availability

No data were used to support this study.
